# A Multistakeholder Approach to the Airport Gate Assignment Problem: Application of Fuzzy Theory for Optimal Performance Indicator Selection

**DOI:** 10.1155/2021/2675052

**Published:** 2021-09-03

**Authors:** Haonan Li, Xu Wu, Yinghui Liang, Chen Zhang

**Affiliations:** ^1^School of Traffic and Transportation, Beijing Jiaotong University, Beijing, China; ^2^China Civil Aviation Engineering Consulting Co., Ltd., Beijing, China; ^3^China Academy of Civil Aviation Science and Technology, Beijing, China

## Abstract

Airport gate assignment performance indicator selection is a complicated decision-making problem with strong subjectivity and difficulty in measuring the importance of each indicator. A better selection of performance indicators (PIs) can greatly increase the airport overall benefit. We adopt a multicriteria decision-making approach to quantify qualitative PIs and conduct subsequent selection using the fuzzy clustering method. First, we identify 21 commonly used PIs through literature review and survey. Subsequently, the fuzzy analytic hierarchy process technique was employed to obtain the selection criteria weights based on the relative importance of significance, availability, and generalisability. Further, we aggregated the selection criteria weights and experts' score to evaluate each PI for the clustering process. The fuzzy-possibilistic product partition *c*-means algorithm was applied to divide the PIs into different groups based on the three selection criteria as partitioning features. The cluster with highest weights of the centre was identified as the very high-influence cluster, and 10 PIs were identified as a result. This study revealed that the passenger-oriented objective is the most important performance criterion; however, the relevance of the airport/airline-oriented and robustness-oriented performance objectives was highlighted as well. It also offers a scientific approach to determine the objective functions for future gate assignment research. And, we believe, through slight modifications, this model can be used in other airports, other indicator selection problems, or other scenarios at the same airport to facilitate policy making and real situation practice, hence facilitate the management system for the airport.

## 1. Introduction

The air transport market has been steadily growing both in the freight and passenger aspects. According to the International Air Transport Association (IATA), in 2019, international passenger traffic climbed 4.1% compared to 2018, down from 7.1% annual growth the year before. Capacity rose 3.0% and load factor edged up 0.8 percentage point to 82.0% IATA [1]. Due to high demand in the air transport industry, many large airports have had to handle hundreds and thousands of flights per day, which greatly stresses airport operations.  Figure 1 depicts the data on gate-constrained airports worldwide, according to WASG [2].

Figure 1 indicates that there has been a consistent increase in the number of gate-constrained airports. According to IATA's reports and estimates, realistically, there could be another 100 airports declared full in 10 years. This poses a significant problem for consumers and the industry, reducing flexibility in scheduling, decreasing the ability to meet passenger demand without serious constraints, and potentially creating nonoptimal flight schedules to fit in with available capacity. Furthermore, 9% of the airports worldwide enable 69% of flights operating in 2019. Based on the IATA statistics reports, the aviation sector is in the midst of a capacity crisis, highlighting the growing relevance of gate assignment.

The airport gate assignment problem (AGAP) has been a popular research topic over the years. Given its nature, AGAP concerns three main stakeholders: the airport operators, the airlines, and the passengers. The airport operator seeks to increase revenues of its shopping facilities and minimise operational costs. Passengers care about convenient boarding, comfortable waiting experience, and ample amenities such as shops and restaurants. As for the airlines, they aim to have easy access to the terminal and short ground times. These differences in stakeholders' perspectives result in a vast range of objectives (Performance Indicators).

When selecting objectives for their algorithms, scholars commonly tend to focus on one or two of the main stakeholders, whereas the on-ground staff must coordinate all three stakeholders' needs. The optimal algorithm can balance the needs of all stakeholders according to the different airports and policies they apply, which further depends on objective selection and weights distribution. In this context, the findings of our study are highly significant.

The review of existing studies indicates that the performance indicator ranking and selection in this field has not received much attention and relevant research is limited. However, it is vital for airport operators and managers to have an overall comprehension of the importance of the PIs. And, it would be informative for scholars when they are designing new algorithms that can be utilized in on-ground operations. In order to fill this research gap, this study aims to investigate which performance indicators affect the on-ground overall benefit the most. The fuzzy analytic hierarchy process (henceforth, fuzzy AHP or FAHP) method coupled with fuzzy *c*-means clustering (FCC) enabled us to rank and categorise the performance indicators (objectives) due to the fuzzy nature of the PIs. With the application of fuzzy AHP, we evaluate each PI under three Selection Criteria—significance, availability, and generalisability—and successfully obtain weights of each PI. Subsequently, the FCC method was employed to divide the PIs across different groups and ranking. The method that we applied in this study not only allowed us to obtain the weights of the PIs but also enabled us to find those PIs that matter the most based on the weights of the cluster centres.

The remainder of this paper is organised as follows. First, an extant literature review of three types of objectives is performed to identify the important performance indicators associated with this problem.  Section 3 elaborates the research method used for the ranking and clustering process of the PIs. This is followed by a discussion of the results and demonstration of our findings. Finally, the summary, conclusion, and recommendations are presented in the last section.

## 2. Literature Review

### 2.1. Identification and Screening of Performance Indicators

The gate assignment problem is a multiobjective optimisation issue in nature because of the multiple stakeholders involved and the numerous and conflicting objectives of each stakeholder. Thus, it is highly necessary to choose the right objectives and prioritise them to facilitate airport operations.

In the early research on the topic, the objective of AGAP was mainly focused on passenger perspectives. Braaksma [3] were the first used total passenger walking distance as the optimizing objective. Since the 1970s, passenger walking distance has become the most commonly used performance indicator in AGAP solution research. Mangoubi and Mathaisel [4] and others used this indicator in their objective functions. In 1984, Babić et al. [5] proposed average passenger walking distance as a new indicator and to supplement passenger walking distance. On the contrary, Chang [6] and Xiao et al. [7] proposed that passenger walking time is more suitable as an indicator especially under mass passenger flow conditions. Furthermore, after consulting with the on-ground staff, they deduced that passenger walking distance can be easily affected by the passenger flow volume, unlike passenger walking time, which made the latter more suitable as a performance indicator. Maharjan and Matis [8] proposed a new indicator—expected passenger discomfort—which was calculated based on walking distance or waiting time and has an overlap with other indicators. Another important passenger-oriented indicator is baggage transport distance, which was proposed by Cheng [9] and Hu and Di Paolo [10]. Passenger waiting time (on the plane) is another indicator mentioned by Yan and Huo [11] and Yan and Tang [12]. Benlic et al. [13] proposed estimated transfer time for passengers as an indicator in 2016. Many such indicators have been examined in previous research, and most of them can be calculated from the aforementioned indicators. Thus, we do not consider them as independent indicators in this paper.

The airport/airline is another important shareholder in this problem. Hence, airport/airline-oriented objectives are a necessity when formulating the objective function. The number of un-gated flight or flights assigned to remote gates is a commonly mentioned indicator in research papers [14–17]. Some researchers [13, 18, 19] used daily towing moves as an independent indicator. Other common indicators include total delay time [20], taxiing time [21, 22], aircraft waiting time (for a gate) [9, 10], and aircraft-gate compatibility [23]. Tang and Wang [24] attempted to maximise the number of arriving flights and the subsequent departing flights assigned to the same gate if served by the same aircraft. Nevertheless, some indicators did not receive much attention, such as total flight-gate preference [15, 25], the fuel consumption of taxiing operations [8], the number of passengers near the shopping facilities [26], and the number of departing flights assigned to short distances to target airline VIP lounges [24].

Due to the nature of air transport, the predetermined assignment plan will be inevitably disturbed by various causes, such as weather conditions, traffic jams, and mechanical failure. Thus, the need for increasing plan robustness has been constantly rising. Also, according to Daş et al. [27], the growing number of articles only considering robustness-related objectives demonstrate the significance of this type of objective. Therefore, we still list robustness as an independent perspective. However, robustness-oriented objectives are more academic and theoretical and are usually hard for on-ground operators to understand or apply. The commonly mentioned indicators under this perspective are idle time [28], variance of the idle time [29–31], expected number of gate conflicts [20], and absolute deviation of new gate assignment from a reference schedule [9, 16]. Other indicators such as expected total semideviation of idle time from buffer time [32] and expected gate conflict cost [33] are mentioned in studies as well.

In summary, there is a vast range of objectives under each perspective. We need to screen some inconsequential indicators before the assessment process to avoid complexity and redundant calculation.

### 2.2. Performance Indicator (PI) Ranking Process

The nature of the performance indicator ranking process is a multicriteria decision-making process. There is a large volume of published papers focused on this issue, and many techniques have been created to make the process as scientific and accurate as possible. The most commonly used and classic decision-making technique is AHP [34]. AHP is a multicriteria decision-making method used to solve complex problems or systems by implementing a pairwise comparison based on the judgement of experts to determine the priority scale of the criteria. It has been applied in many areas for its convenience and efficiency in measuring multiple criteria. However, through years of development and research, scholars have proposed the concern that classic AHP cannot reflect the actual human logic in which uncertainty and subjectivity may occur with the factor comparisons [35].

To solve this problem, the classic AHP method has been improved by applying a fuzzy method [36]. Another method, the entropy weight method (EWM), is an efficient comprehensive index evaluation method; however, this method requires an existing efficiency result of each criterion to complete the process, which is extremely difficult to ask airports to do so. Thus, the EWM is not suitable for the gate assignment PI ranking process. There are also other improved methods that are meant to overcome the drawbacks of classic AHP. Interval multiplicative preference relation is widely used in decision-making [37], and the fuzzy best-worst method is also proposed as an improved method [38, 39].

One significant feature of the PIs in AGAP is the fuzziness. A large number of the PIs are difficult to evaluate quantitively, thereby making it hard to determine their relative importance quantitively. Thus, we introduce fuzzy math into the PI ranking process as a relatively optimal solution. Fuzzy AHP is an improved AHP method. It overcomes the main drawback of classic AHP, such as incapable of reflecting expert's opinion using crisp ratings. And, it can maintain the reliability of the classic AHP at the same time. Expert's opinion regarding PIs in AGAP are commonly varied and uncertain. FAHP can allow uncertainty to a certain extent without undermining the validity, which is why we chose this method. Further, the classic AHP method requires experts to fill out a pairwise comparison matrix, which is painstaking. Although filling out a questionnaire is vital for the retrieval of the data, an exhausting survey experience may compromise the quality of the data. An adapted version of questionnaire must be designed to shorten the filling-out time. The improved fuzzy AHP method [40], coupled with trapezoidal fuzzy numbers (TraFN), is adopted to reflect actual human logic. FAHP is used to estimate the weights of the three selection criteria for the corresponding PI [41]. Moreover, the improved FAHP can greatly reduce the time required to fill out a questionnaire without compromising the quality.

### 2.3. PI Selection and Clustering

During a PI selection process, there usually are many more PIs than we need. Even after obtaining the rank of PIs, the problem of partitioning or dividing them into groups remains. Randomly partitioning or choosing based on the scholars' own opinions may leave out some important PIs. Thus, a clustering method based on the ranking results is implemented.

Clustering algorithms are part of a large machine-learning family with different starting points and criteria. Due to the goal of this clustering method is to distinguish those PIs that have more impact on the on-ground operation from other inconsequential PIs, partitioning-based algorithms stand out for not only being robust, scalable, and simple but also easy to understand and meeting our needs.

Hence, partitioning-based algorithms are most suitable in this case. *K*-means clustering [42] is the most commonly used partitioning-based algorithm and is known as hard clustering. It is a machine learning process to partition elements into different clusters based on their similarity. Many researchers [43, 44] have used *K*-means clustering as an efficient tool for image segmentation. In these studies, the common approach involves using the RGB index of each pixel as the feature and evaluating similarity and partition images based on it. There is a similarity between image segmentation and our PI selection. The RGB index is a three-dimension vector same as our crisp local weights. Analogously, the three selection criteria are considered as the features for the clustering algorithm.

However, as datasets usually cannot be divided into distinct clusters, it is irrational to categorise every PI into distinct clusters. In this case, a soft clustering method emerged, known as fuzzy *c*-means clustering (FCC). Similar to *K*-means clustering, the FCC method is widely used in image segmentation [45, 46]. Cao et al. [47] applied FCC for providing sensor deployment strategy for indoor environment control, thus proving that application of FCC can facilitate the decision-making process. The results of FCC indicate the cluster membership of each data point, unlike *K*-means, which directly divides data points into distinct clusters. Based on the specific problem, it is possible to adjust the fuzziness of the partition through parameters. The FCC method offers a more flexible clustering result which made this approach suitable for gate assignment PI selection. However, traditional FCC has high outlier sensitivity. Gosztolya and Szilagyi [48] proposed an improved FCC algorithm by including probabilistic and possibilistic terms and combining them via multiplication to achieve better partitions. This is called the fuzzy-possibilistic product partition *c*-means algorithm (FPPPCM), and it can reduce the number of parameters while efficiently reject the effect of outliers. Hence, FPPPCM is suitable and robust for gate assignment PI clustering.

Indicators' ranking is a common procedure in a managerial problem. However, ranking only tells us about the importance of the indicators not how to choose then. In common cases, indicators are still subjectively chosen. But with the clustering technique, it offers a data-driven method to select the indicators. FAHP is selected for its ability to comply with the human logic and its reliability. FPPPCM is applied for its efficiency and insensibility of outliers. A technique that we proposed combined both advantages together allowing us to rank and choose the most suitable PIs without subjectivity.

## 3. Methodology

This research conducts FAHP and FPPPCM to determine the relative influence of the performance criteria and indicators of the gate assignment problem.

This research consists of four phases which are illustrated as in Figure 2.

### 3.1. Fuzzy Theory

In this study, fuzzy theory is applied to assess multiple predetermined criteria with a nature of uncertainty and vagueness. As experts' opinions are certain within an interval regarding PIs in AGAP, we adopted TraFN.

The membership of a fuzzy number (Figure 3) is defined as follows:

(1) $$\begin{array}{c} u\left(x\right)=\left\{\begin{array}{cc} 0, & \left(x<m_{1}\right),\\ \frac{x-m_{1}}{m_{2}-m_{1}}, & \left(m_{1}\leq x\leq m_{2}\right),\\ 1, & \left(m_{2}\leq x\leq m_{3}\right),\\ \frac{m_{4}-x}{m_{4}-m_{3}}, & \left(m_{3}\leq x\leq m_{4}\right),\\ 0, & \left(x>m_{4}\right). \end{array}\right. \end{array}$$

The trapezoidal fuzzy number is denoted as *M*_1_=(*a*_1_, *b*_1_, *c*_1_, *d*_1_), and operational laws that will be used later are as follows:

(2) $$\begin{array}{c} \left(1\right)\;\left(a_{1},b_{1},c_{1},d_{1}\right)⊕\left(a_{2},b_{2},c_{2},d_{2}\right)=\left(a_{1}+a_{2},b_{1}+b_{2},c_{1}+c_{2},d_{1}+d_{2}\right),\\ \left(2\right)\;\left(a_{1},b_{1},c_{1},d_{1}\right)⊗\left(a_{2},b_{2},c_{2},d_{2}\right)=\left(a_{1}a_{2},b_{1}b_{2},c_{1}c_{2},d_{1}d_{2}\right),\\ \left(3\right)\;{\left(a_{1},b_{1},c_{1},d_{1}\right)}^{-1}=\left(\frac{1}{d_{1}},\frac{1}{c_{1}},\frac{1}{b_{1}},\frac{1}{a_{1}}\right). \end{array}$$

According to the theory mentioned above, the membership function of linguistic scales is illustrated in Table 1:

### 3.2. Defining Selection Criteria and PI Identification

After conducting a consultation with scholars and experts, three selection criteria were established: (1) significance, (2) availability, and (3) generalisability.

Instead of scoring the PI using numbers, a linguistics assessment was performed using words in natural languages, which is useful to obtain opinions. In this study, we coupled TraFN with a linguistic scoring scheme, which allows us to assess the PIs as illustrated in Table 2.

Based on an extensive literature review, we identified and screened 21 performance indicators under three performance criteria, which are considered possibly influential to the on-ground operations.  Table 3 shows the definition and resource of each indicator.  Figure 4 demonstrates the hierarchical structure of the process.

### 3.3. Survey Implementation

We designed a survey questionnaire to collect expert opinions on significance, availability, and generalisability of the indicators. The questionnaire comprised several sections. The first section described the purpose of this survey, collected opinions about current algorithm applications, and provided instructions about filling out the questionnaire. The second section asked respondents to compare the three selection criteria in pairs to determine their relative importance. In the third section, we asked respondents to score the three criteria for each indicator. The last section enabled respondents to suggest indicators that we had not mentioned and score them as per the three criteria.

12 airports were selected based on the traffic and the locations. As shown in Figure 5, selected airports covered main parts of China. However, only the busiest airports would face the gate-constrained problem, and east of China is more developed than the west, and this is why these airports mainly located in east and middle. As we can see in Table 4, all the airports we selected are on top 20 of China, and 2 of them are on top 10 busiest airports in the world [49], which makes our survey not only convincing but also representative. Beijing Daxing International Airport is newly opened mega airport in China. Based on its status in China, we believe it will enhance our survey results if it is included. Survey was sent to the liaison team that constituted of staff and experts of the airport or relevant area. A wide range of respondents is covered, of which 42% are on-ground operators, 33% are executive officers, and 25% are researchers. While all respondents have a bachelor's degree, 41.6% also have a Master's or a higher degree. All the respondents have at least a three-year experience, which is considered to be able to balance three stakeholders' opinion.

### 3.4. Fuzzy-Possibilistic Product Partition *C*-Means Clustering (FPPPCM)

FCC is used as an efficient tool to divide data points into different groups. This method is also known as soft clustering. Unlike hard clustering, such as *K*-means, the FCC allows one piece of data to belong to two or more clusters, which is more in accordance with reality. The degree of membership indicates the level of association of the element within the formed cluster, which is a unique feature of FCC. In order to eliminate the outlier sensitivity of the original FCC model, FPPPCM [48] is adopted.

We used the statistical software *R* to conduct the FPPPCM analysis.

The FPPPCM algorithm is based on the minimisation of the following objective function:

(3) $$\begin{array}{c} J_{\text{FPPPCM}}=\sum_{i=1}^{N}\sum_{j=1}^{C}u_{ij}^{m}\left[t_{ij}^{p}{\left\|x_{i}-y_{j}\right\|}^{2}+{\left(1-t_{ij}^{p}\right)}^{p}\eta_{j}\right],\;1\leq m,p<\infty , \end{array}$$

where *m* is the degree of fuzziness, commonly between 1.25 and 2, a higher value of which leads to higher fuzziness, *p* is the possibilistic exponent, *η*_*i*_ is the conventional penalty terms of the possibilistic partition, which is used to control the variance of the clusters, *u*_*ij*_ is the degree of membership of *x*_*i*_ in the cluster *j*, *x*_*i*_ is the *i*^th^ of three-dimensional data vector (significance, availability, and generalisability), *y*_*j*_ is the three-dimensional centre of the cluster, *∗* is any norm expressing the similarity between any measured data and the centre, *N* is the number of PIs, and *C* is the number of clusters.

*t*_*ij*_ denotes typicality values, which are used to describe how compatible the input weight vectors are with clusters represented by the calculated cluster prototype:

(4) $$\begin{array}{c} t_{ij}^{*}={\left[1+{\left(\frac{{\left\|x_{i}-y_{j}\right\|}^{2}}{\eta_{j}}\right)}^{\left(1/\left(p-1\right)\right)}\right]}^{-1}. \end{array}$$

In this study, the elbow method is adopted to determine the number of the cluster. The elbow method depicts an increase in the number of clusters with a decrease in the within group sum of squares. The result is shown in Figure 6.

Euclidean distance is used to express similarity between the PI and the cluster centre. Thus, the degree of membership and the cluster centres can be calculated as follows:

(5) $$\begin{array}{c} u_{ij}^{*}=\frac{{\left[t_{ij}^{p}{\left\|x_{i}-y_{j}\right\|}^{2}+{\left(1-t_{ij}\right)}^{p}\eta_{j}\right]}^{\left(-1/\left(m-1\right)\right)}}{\sum_{k}^{C}{\left[t_{ik}^{p}{\left\|x_{i}-y_{k}\right\|}^{2}+{\left(1-t_{ik}\right)}^{p}\eta_{k}\right]}^{\left(-1/\left(m-1\right)\right)}},\;\forall i\in \left[1,N\right],\forall j\in \left[1,C\right],\\ y_{j}^{*}=\frac{\sum_{i}^{n}u_{ij}^{m}t_{ij}^{p}x_{i}}{\sum_{i}^{n}u_{ij}^{m}t_{ij}^{p}},\;\forall j\in \left[1,C\right]. \end{array}$$

At the beginning of the algorithm, random centres are selected, and new centres can be updated through the objective function and the aforementioned equation. The iteration will stop when max_*ij*_|*u*_*ij*_^*k*+1^ − *u*_*ij*_^*k*^| < *ε*, where *ε* is a termination criterion between 0 and 1, whereas *k* is the iteration step.

The FPPPCM analysis is conducted with these parameters: centres = 3, *m* = 1.25, *p*=2, and *η*_*j*_ = 1. Centres are obtained from the elbow method, and *m*, *p*, and  *η*_*j*_ are default parameters. The procedure of FPPPCM is given in Algorithm 1.

### 3.5. Fuzzy AHP Process and PI Selection

Notations that will be used are listed in Table 5.

  Step 1. Forming fuzzy pairwise comparison matrix: in the second section of the questionnaire, *X* number of respondents (experts) rated the relative importance between three selection criteria using the rating scheme listed in Table 1. Based on the results, we established a fuzzy pairwise comparison matrix (*R*^*～X*^).
  Step 2. Matrix consistency test: after the establishment of the fuzzy pairwise comparison matrix, the consistency must be assessed using the consistency ratio (CR), which is proved that can be used the same test method in classic AHP [50, 51]:
  (6) $$\begin{array}{c} \text{CR}=\frac{\text{CI}}{\text{RI}},\\ \text{CI}=\frac{\lambda_{\max}-n}{n-1},\;n=3, \end{array}$$
where RI is the random index, as shown in Table 6, CI is the consistency value, *λ*_max_ is the largest eigenvalue, and *n* is the dimension. Only if the matrix passed the consistency test, then we can proceed. Otherwise, adjust the matrix until it passes.
  Step 3. Transforming fuzzy pairwise comparison matrix into fuzzy number matrix: by using Table 1, the fuzzy rating can be transformed into fuzzy numbers to obtain the new fuzzy number matrix (*A*^∼*X*^) from *R*^*～X*^, where ${\tilde{a}}_{ij}=\left[{\left(a_{ij}\right)}_{a},{\left(a_{ij}\right)}_{b},{\left(a_{ij}\right)}_{c},{\left(a_{ij}\right)}_{d}\right]$, for further calculation.
  Step 4. Fuzzy local weights calculation: the normalised geometric mean [51] is used to calculate the weights of each criterion (*W*_*i*_). Thus, it is used to calculate four elements of the TraFN, respectively:
  (7) $$\begin{array}{c} W_{i}=\left[{\left(w_{i}\right)}_{a},{\left(w_{i}\right)}_{b},{\left(w_{i}\right)}_{c},{\left(w_{i}\right)}_{d}\right],\\ w_{i}=\frac{\sqrt[{3}]{a_{i1}\times a_{i2}\times a_{i3}}}{a_{i1}+\sqrt{a_{i1}\times a_{i2}}+\sqrt[{3}]{a_{i1}\times a_{i2}\times a_{i3}}}. \end{array}$$
  Step 5. Local weights aggregation: the final local weights of each criterion are taken as the arithmetic mean:
  (8) $$\begin{array}{c} {\tilde{\bar{W}}}_{i}=\frac{\sum_{1}^{X}{\tilde{W}}_{i}^{X}}{X}. \end{array}$$
Experts also scored each PI in the third section of the questionnaire. Thus, we aggregate the score $\left({\tilde{S}}_{i}\right)$ with the fuzzy weights of each criterion $\left({\tilde{\bar{W}}}_{i}\right)$, using the equation below to obtain the fuzzy local weights of each indicator for subsequent ranking and clustering:
  (9) $$\begin{array}{c} {\tilde{\omega }}_{i}={\tilde{\bar{W}}}_{i}\times \left(\sum_{1}^{X}{\tilde{S}}_{i}^{X}\right). \end{array}$$
  Step 6. Defuzzification: the arithmetic means of the TraFN are considered as the crisp local weights:
  (10) $$\begin{array}{c} \omega_{i}=\frac{{\left({\tilde{\omega }}_{i}\right)}_{a}+{\left({\tilde{\omega }}_{i}\right)}_{b}+{\left({\tilde{\omega }}_{i}\right)}_{c}+{\left({\tilde{\omega }}_{i}\right)}_{d}}{4}. \end{array}$$
  Step 7. PI clustering: the FPPPCM analysis is performed to obtain clustering results.
  Step 8. Obtain global weights: after the clustering analysis, the ranking process is conducted based on the weights of the cluster centre. Further, we normalise local weights of selected PIs to obtain the global weights:

(11) $$\begin{array}{c} {\text{GW}}_{i}=\frac{\omega_{i}}{\sum_{i}^{n}\omega_{i}},\;n=\text{number of elements in very high influence cluster}. \end{array}$$

## 4. Results and Discussion

The final results and figures are demonstrated in Table 7 and Figure 7. The preliminary objective of this study is to identify the PIs that affect the on-ground operations the most. Thus, the ranking of the PIs will be discussed in this section. The total weights were calculated as the sum of the three selection criteria weights, and the ranking index was normalised.  Table 8 presents the fuzzy weights of three selection criteria. Table 7 demonstrates the ranking and global weights of PIs that were categorised in very high-influence clusters.  Table 9 is weights of cluster centres and the category each belongs to. And, Table 10 shows the ranking of each performance criterion based on the average weights.  Figure 7(a) demonstrates the selecting efficiency of all the performance criteria and scatter plots of all the PIs are demonstrated in Figure 7(b). A detailed literature review, summarised in Table 3, enabled us to identify the 21 indicators that were evaluated under these criteria.

### 4.1. Passenger-Oriented Objective

In civil aviation, passengers' satisfaction plays a significant role in airport operations. According to the results in Tables 7 and 10, there are four PIs belonging to the very high-influence cluster, and passenger-oriented objectives received the highest average weights, making it the most important criterion. Among all the indicators in this objective, passenger walking time ranks the highest. Chang [6] mentioned that passenger walking time has a significant impact on passenger comfort. Furthermore, Teng et al. [52] in their research on metro station congestions based on passenger time perceptions proved that passenger walking time is an important indicator of passenger satisfaction and has a great influence on passengers' perception of congestion. Hence, it is no surprise that passenger walking time ranks second in our findings.

Baggage transit distance is considered as another factor affecting passenger comfort as it impacts the time that passengers wait for their luggage [9]. One interesting finding of our ranking is that baggage transit distance, which did not receive as much attention in previous research [53], has a moderately high weight, with the rank of the third in the chart. Thus, this should be considered as an important indicator in future research, when it comes to modelling.

Another interesting result is that, while average passenger walking distance received a high weight, with the fourth rank in the chart, it did not outrank passenger walking time. The existing study [4, 10] found that passenger walking distance has a direct impact on passenger satisfaction. Passenger walking distance usually means the sum of the distance walked by passengers between two adjacent boarding activities in a day. However, based on our results, the reason for the low rank is due to the significance weight of the PI. After consulting with on-ground operators about the results, the reasons that we gathered are that (1) passenger walking distance can be easily influenced by the size of the airport; (2) passenger walking time can be more intuitively perceived to value the congestion of the airport.

Another indicator that received a high weight is passenger waiting time on the plane. According to Yan and Huo [11], waiting on the plane can significantly undermine the satisfaction of passengers because there are no shops or recreational activities to while away the waiting time.

Notably, four of the five passenger-oriented PIs are categorised under the very high-influence cluster, thereby confirming that the passenger represents the most essential criterion among the three performance criteria. It is surprising to note that estimated passenger transfer time did not receive much attention among the respondents who completed the questionnaire. This could be because the airport operator intends to set aside enough time for passengers to visit the shopping facilities to increase potential commercial revenues.

### 4.2. Airport/Airline-Oriented Objective

The airport/airline-oriented objective is the second important criterion of airport overall benefit. Unlike the passenger-oriented objective, which focuses on improving passenger satisfaction, the airport/airline-oriented objective mainly aims to reduce cost and increase efficiency. The result shows that the number of flights assigned to remote gates is the most important one among all the other indicators. Drexl and Nikulin [25] reported that assigning flights to remote gates needs bus transfer operations, which may increase the connection time and can thus be hardly regarded as desirable. Moreover, assigning flights to remote gates increases the baggage transfer distance, which can both undermine passenger satisfaction and the airport's operational costs. These results are in line with previous studies [9, 15–17, 24] that state that the use of remote gates is highly undesirable. In fact, under the Federal Aviation Administration (FAA) Regulations, all US airports are forbidden to assign their flights to remote gates. However, in most countries, we do not see such strict regulations that can increase operational difficulties.

Nevertheless, it can be seen from Table 8 that there are quite a few indicators in this criterion that belong to the very high-influence cluster with daily towing moves, total flight delay, and taxiing time ranking fifth, sixth, and seventh, respectively. We define moving an airplane between two positions as a tow. Towing activities require time and resources (towing tractors). Dorndorf et al. [18] and Dijk et al. [54] stated that too many towing moves can significantly increase the cost, in terms of time and money, which is undesirable for both airport authorities and passengers. In this context, it is not a surprise that daily towing moves received a high weight. The noteworthy result is that the rank of total flight delay is not so high as expected. This may be explained by the fact that 46.49% of the flight delays in China last year was due to weather conditions [55], which despite being an uncontrollable factor, needs to be accommodated and not avoided. According to Kim et al. [21], longer taxiing time implies more local emissions and noise. Considering the objective of reducing operational costs and environmental impact, taxiing time is an important factor that should be of concern to researchers.

As shown in Table 7, there are many other indicators under this criterion. These are inconsequential compared with the ones mentioned above. However, the number of consecutive flights is much less inconsequential than expected, even though it was categorised in the very high-influence cluster. Tang and Wang [24] pointed out that using one aircraft to serve two adjacent flights can also reduce the towing movements and increase ground service convenience and efficiency, thereby reducing the shift in the ground service staff for the two flights and subsequently, the flight delay. Based on the resultant weight, one possible explanation for the low rank can be that it will increase difficulty in operations and would be hard to promote in all the airports. Another interesting result is that aircraft-gate size compatibility received a low rank (not being categorised in very high-influence cluster). This may be because the on-ground staff only need the gate size to be sufficiently usable for the aircraft and are not pursuing 100% compatibility.

### 4.3. Robustness-Oriented Objective

Like all other airport operations, gate assignment could be inevitably disrupted by various unexpected situations. Hence, gate planners need to take robustness into account as well. In common cases, researchers use either idle-time- or gate-conflict-based approaches to achieve robustness of the schedules.

The ranking results are striking because all the indicators under this criterion did not receive much attention as we had presupposed. The variance of idle time is the only PI that is categorised in very high-influence cluster under this criterion. Bolat [28], Daş [26], and Deng et al. [56] agree that a better balance of idle time allows gate assignment plans to cope with more time variations of arrival and departure flights.

Other indicators under this criterion, such as idle time, number of gate conflicts, and absolute deviation of new gate assignment from a reference schedule, are considered as inconsequential indicators. This was found to be due to the application difficulty of these indicators. All these indicators received low generalisability weights compared to others, which means that most of the gate planners consider these indicators to be hard to achieve or promote in a wide range of airports.

However, it does not mean robustness is not important. It shows the differences in priorities between researchers and on-ground staff, which is an important issue for future research and a potential practical implication of the study. Future work should find a balance between theoretical objectives and practical objectives, to obtain a suitable objective function for mathematical modelling.

### 4.4. Application of the Proposed PI Selection Process

Selected indicators that can demonstrate the higher airport overall benefit are usually varied between different airports even different scenarios of the same airport, for the airport policies, the regulation of the Aviation Administration, and the definition of the overall benefit of the specific airport scenario are different. However, currently, there is no systematic way for the airport to select the indicators and distribute adequate weights to them. The process we proposed filled in this gap by offering a scientific way to select the indicators and distribute the weight.

## 5. Conclusion

### 5.1. Conclusions and Limitations

This study identified 21 common PIs mentioned in previous research. Through the PI selection process, we determined 10 PIs that have a very high influence on the on-ground operation: 5 under airport/airline-oriented, 4 under passenger-oriented, and 1 under robustness-oriented performance criteria.

The method that is employed in this study is a highly suitable approach for such a problem. The FAHP method allowed us to obtain weights and rank of the PIs, and the FPPPCM algorithm enabled us to partition and select relevant PIs.

In general, while it seems that some results comply with our common knowledge and practical understanding of the importance of the PIs, our analysis brought out certain noteworthy issues as well. However, they also demonstrate a difference in opinion and priorities between scholars and on-ground staff. For example, baggage transit distance has a surprisingly high rank, while few papers mentioned it or adopted it as an objective. The accordance with previous studies proved that our research is not only reliable but also has shed new light on AGAP objective selection.

One limitation of this paper is that the number of respondents may have an impact on the analysis results. And, due to the constantly changing operation environment, this paper only reflects the current static situation. While three performance criteria are considered, there may exist more performance criteria that can influence the airport overall benefit.

### 5.2. Managerial and Theoretical Implications

Apart from AGAP, many other transport management indicator selection problems require considering the quantitative aspect, and the approach proposed in this paper better solves the problem combining quantitative and qualitative perspective and provides these implications and applications:

1. Future practice in this field may find this research useful for providing scientific proof for objective selection. Especially, when scholars are solving gate assignment problem applying the deep learning algorithm or other artificial intelligence algorithms, the selection of the objective functions can significantly affect the results and the efficiency of the algorithm.
2. The aforementioned approach can help on-ground operators and airport managers to choose appropriate performance indicators during policy-making and practice.
3. This approach can be used in other indicator selection problems, other countries, and different scenarios at the same airport with slight modifications.

In future, we may consider more factors not only focusing on operational aspects but also other aspects such as carbon emissions or other environmental factors. More refined methods [37] and consistency tests [57, 58] can be used to improve the reliability of the clustering algorithm. And, we may consider using new techniques to adapt the problem into group decision-making [59, 60]. We recommend this study as a starting point. With the development of techniques, ideally we can correctly select out the most suitable PIs for each distinct airport to better facilitate on-ground operation.

## Figures and Tables

**Figure 1:** Gates-constrained airports worldwide.

**Figure 2:** PI selection process for the gate assignment problem.

**Figure 3:** The membership of a fuzzy number.

**Figure 4:** Hierarchical structure of the PI selection.

**Figure 5:** Distribution of surveyed airports.

**Figure 6:** The elbow method.

**Figure 7:** (a) Selection efficiency. (b) Scatter plots of PIs in different clusters. Note: the size of the bubble indicates the final weights of each PI, and the colour indicates the cluster it belongs to. The corresponding cluster category is in Table 8.

**Algorithm 1:** Procedure of FPPPCM.

**Table 1:** Membership function of linguistic scales.

Degree of importance	Fuzzy rating	TraFN
Equally important	1	(1, 1, 1, 1)
Intermediate	2	(1, 1.8, 2.2, 3)
Weakly more important	3	(2, 2.8, 3.2, 4)
Intermediate	4	(3, 3.8, 4.2, 5)
Important	5	(4, 4.8, 5.2, 6)
Intermediate	6	(5, 5.8, 6.2, 7)
Very important	7	(6, 6.8, 7.2, 8)
Intermediate	8	(7, 7.8, 8.2, 9)
Extremely more important	9	(9, 9, 9, 9)

**Table 2:** Linguistic scoring scheme for selection criteria.

Linguistic scoring	TraFN	Selection criteria		
		Significance	Availability	Generalisability
Low	(0, 0.1, 0.4, 0.5)	The PI is insignificant and may not affect airport operation assessment if not included	The PI is hard to measure or data is hard to obtain	The application of PI is difficult in most of the airports

Medium	(0.25, 0.35, 0.65, 0.75)	PI is significant and may improve airport operation assessment	PI can be measured or data is easily accessible	The application of PI asks for certain requirements of the airport, but still applicable

High	(0.5, 0.6, 0.9, 1)	PI is highly significant; the overall benefit assessment may not be reliable if not included	PI can be easily measured, and the data is easy to obtain	PI can be easily applied in most of the airports

**Table 3:** Performance indicators for AGAP.

Performance criterion	Performance indicator	Source	Notes
Passenger-oriented objectives	Passenger walking time	[6, 7]	
	Average passenger walking distance	[3–5]	
	Baggage transit distance	[9, 10]	
	Passenger waiting time	[11, 12]	
	Estimated passenger transit time	[13]	

Airport/airline-oriented objectives	Number of flights assigned to remote gates	[14–17]	Or known as un-gated flight in some research papers
	Daily towing moves	[13, 18, 19]	
	Total flight delay	[20]	
	Taxiing time	[21, 22]	
	Aircraft waiting time (for a gate)	[9, 10]	
	Number of consecutive flights	[24]	Number of arriving flights and the subsequent departing flights assigned to the same gate, if served by the same aircraft
	Total flight-gate preferences	[15, 25]	
	Fuel consumption of taxiing operations	[8]	
	Number of passengers at gates close to shopping facilities	[26]	
	Aircraft gate size compatibility	[23]	
	Number of departing flights assigned close to the target airline VIP lounges	[24]	
	Number of flights assigned close to customs	[24]	

Robustness-oriented objectives	Variance of the idle time	[29–31]	
	Absolute deviation of new gate assignment from a reference schedule	[9, 16]	
	Expected gate conflicts	[20]	
	Idle time	[28]	

**Table 4:** Statistics of surveyed airports.

Name	City	Passenger enplaning and deplaning^*∗*^	Taking off and landing^*∗*^	Ranking in China (based on passenger traffic)	Top 10 busiest airports in the world^*∗∗*^ (yes/no)
Beijing Capital International Airport	Beijing	100,013,642	594,329	1	Yes

Shanghai Pudong International Airport	Shanghai	76,153,455	511,846	2	Yes

Guangzhou Baiyun International Airport	Guangzhou	73,378,475	491,249	3	Yes

Shenzhen Baoan International Airport	Shenzhen	52,931,925	370,180	5	No

Shanghai Hongqiao International Airport	Shanghai	45,637,882	272,928	8	No

Chongqing Jiangbei International Airport	Chongqing	44,786,722	318,398	9	No

Hangzhou Xiaoshan International Airport	Hangzhou	40,108,405	290,919	10	No

Zhengzhou Xinzheng International Airport	Zhengzhou	29,129,328	216,399	12	No

Wuhan Tianhe International Airport	Wuhan	27,150,246	203,131	14	No

Changsha Huanghua International Airport	Changsha	26,911,393	196,213	15	No

Qingdao Liuting International Airport	Qingdao	25,556,278	186,500	16	No

Beijing Daxing International Airport	Beijing	—	—	—	No

^*∗*^Based on collected data in 2019. ^*∗∗*^According to ACI, 2020.

**Table 5:** Notations.

Notations	Definitions
*X*	Number of respondents (experts)
*R*	Fuzzy pairwise comparison matrix
CI	Consistency value
RI	Random index
*n*	The number of dimensions (significance, availability, and generalisability)
CR	Consistency ratio
*A*	Transformed fuzzy pairwise comparison matrix
*W*	Weights of each criterion
*S*_*i*_	Aggregated expert score of criterion *i*
*ω*	Crisp local weights of the PI
GW	Global weights of the PI in selected group

**Table 6:** Random index.

*n* (dimension)	1	2	3	4	5	6
RI	0	0	0.52	0.89	1.12	1.26

**Table 7:** Ranking of very high-influence clusters.

PI	SIG	AVA	GEN	GW	Criterion
Number of flights assigned to remote gates	3.4566	4.0351	3.2843	0.1130	Airport/airline
Passenger walking time	3.2137	3.5071	3.3443	0.1055	Passenger
Baggage transit distance	3.2137	3.5071	2.9786	0.1017	Passenger
Average passenger walking distance	2.7228	3.6391	3.2249	0.1005	Passenger
Daily towing moves	3.2137	3.5071	2.8542	0.1004	Airport/airline
Total flight delay	3.4566	3.1084	2.8567	0.0988	Airport/Airline
Taxiing time	3.0897	3.3751	2.7323	0.0964	Airport/airline
Passenger waiting time	3.2112	3.2404	2.7372	0.0963	Passenger
Variance of the idle time	3.0922	3.2430	2.6104	0.0938	Robustness
Number of consecutive flights	3.0897	3.2404	2.6104	0.0937	Airport/airline

*Note.* PI = performance indicator; SIG = significance; AVA = availability; GEN = generalisability; GW = global weight.

**Table 8:** Selection criteria fuzzy weights.

Selection criteria	Fuzzy weights			
Significance	0.4772	0.4891	0.4942	0.5031
Availability	0.5039	0.5335	0.5420	0.5542
Generalisability	0.4790	0.4904	0.4959	0.5049

**Table 9:** Cluster centres.

Cluster	SIG	AVA	GEN	Total weights	Ranking index	Category
1	2.4749	2.707	2.4836	7.6655	0.8583	Moderate
2	3.0922	2.8446	2.735	8.6718	0.9057	High
3	3.2137	3.5071	2.8542	9.575	1	Very high

**Table 10:** Performance criteria ranking.

Performance criteria	Average weights	Rank
Passenger-oriented objectives	9.6350	1
Airport/airline-oriented objectives	9.5820	2
Robustness-oriented objectives	8.9456	3

## Data Availability

The data used to support the findings of this study are available from the corresponding author upon request.
